The article "Analysis of Efficacy, Safety, and Prognostic Factors of mFOLFOX6 Regimen Combined with Cetuximab and Simvastatin in the Treatment of K-RAS Mutant Colorectal Cancer" was retracted in 2023. Reasons: unreliable results or conclusions; concerns about the data; concerns about the peer review; concerns about the citations.

# Analysis of Efficacy, Safety, and Prognostic Factors of mFOLFOX6 Regimen Combined with Cetuximab and Simvastatin in the Treatment of K-RAS Mutant Colorectal Cancer

**DOI:** 10.1155/2021/2280440

**Published:** 2021-09-13

**Authors:** Guodong Li, Jiangang Liu

**Affiliations:** Department of Gastrointestinal Surgery, The Second Affiliated Hospital of Shandong First Medical University, Tai'an 271021, Shandong, China

## Abstract

Colorectal cancer (CRC) is one of the most common malignant tumors with high morbidity and mortality. The early symptoms are latent, and most patients are in the middle or late stage when they are diagnosed. The best opportunity for surgery has been lost, and surgical resection has failed to achieve good results. In clinical practice, targeted therapy or chemotherapy is usually the main treatment. The mFOLFOX6 regimen is a standardized regimen for the treatment of advanced CRC. The main drugs in this regimen are oxaliplatin and 5-fluorouracil (5-FU). Patients with advanced CRC combined with standard chemotherapy regimens can achieve a higher resection rate of liver metastases in unresectable patients, which can achieve significant survival improvement. Therefore, in this study, oxaliplatin + calcium folinate + 5-Fu + mFOLFOX6 regimen was combined with cetuximab and simvastatin to treat CRC patients, and the clinical efficacy and prognosis were analyzed, as well as the prognostic factors. The results showed that the addition of simvastatin on the basis of conventional mFOLFOX6 regimen combined with cetuximab chemotherapy could effectively improve the efficacy, reduce the total incidence of adverse reactions, improve the overall survival rate, and prolong the overall survival time of patients. Pathological grade and peritoneal metastasis were the factors affecting the mean survival time of CRC patients.

## 1. Introduction

Colorectal cancer (CRC) is one of the most common malignant tumors in China, with a high morbidity and mortality rate [1, 2]. With economic development and changes in dietary structure, the incidence of CRC is increasing year by year [3, 4]. The symptoms of this disease are latent in the early stage, and most patients are already in the middle or late stage when the disease is diagnosed. Patients have lost the best opportunity for surgery, and surgical resection can no longer achieve good results. In clinical practice, targeted therapy or chemotherapy is usually the main method [5, 6]. Epidermal growth factor receptor (EGFR) is overexpressed in many tumor tissues and participates in the proliferation, differentiation, and apoptosis of tumor cells [7, 8]. Kirsten rat sarcoma viral oncogene homolog (K-RAS) encodes RAS protein, which plays an important role in tumor formation, cell proliferation, cell migration, tumor diffusion, and angiogenesis. K-RAS gene is a downstream signaling molecule of EGFR. When K-RAS gene is mutated, its expression is not regulated by EGFR signal, which leads to abnormal proliferation and metastasis of tumor cells, and then leads to resistance of patients to EGFR inhibitor drugs [9–12]. In recent years, with the advent of oxaliplatin and irinotecan, new modes of administration, new chemotherapy drugs, and new combination regimens, new breakthroughs have been made in the treatment of metastatic CRC, especially in the aspect of molecular targeted therapy [13, 14]. Patients with advanced CRC combined with standard chemotherapy regimens can achieve a higher resection rate of liver metastases in unresectable patients, which can achieve significant survival improvement. Therefore, this study treated CRC patients with oxaliplatin + calcium folinate + 5-fluorouracil (5-FU) + mFOLFOX6 combined with cetuximab and simvastatin and analyzed the clinical efficacy for clinical reference. Specific research studies are as follows.

## 2. Materials and Methods

### 2.1. Patients

A total of 116 CRC patients with K-RAS gene mutation were admitted to our hospital from March 2015 to March 2017. Among them, 64 were males and 52 were females, aged from 31 to 75 years old, with an average age of (50.18 ± 9.48) years old: 82 patients in the left half rectum, 34 patients in the right half colon; 80 patients were moderately or highly differentiated, 36 patients were poorly differentiated; 12 patients had peritoneal metastasis, and 104 patients had no peritoneal. Inclusion criteria: CRC was diagnosed by histopathological examination [15]. The K-RAS gene test showed K-RAS gene mutation; there is at least one detectable lesion; the expected survival time is ≥3 months. Exclusion criteria: combined with other malignant tumors; patients with damage to the heart, liver, and other organs; presence of oxaliplatin, 5-FU, cetuximab, and simvastatin drug allergy; pregnant or lactating women; combined with mental disorders cognitive dysfunction; and patients with follow-up loss. According to chemotherapy methods, they were divided into the control group (*n* = 58) and the observation group (*n* = 58), and there were no statistically significant differences in age, gender, tumor location, pathological grade, and other general clinical data between the two groups (*P* > 0.05), but with comparability, as given in Table 1.

### 2.2. Treatment Methods

#### 2.2.1. Control Group

The control group was treated with mFOLFOX6 combined with cetuximab. On the first day, 85 mg/m^2^ of oxaliplatin (Zhejiang Haizheng Pharmaceutical Co., Ltd.) was intravenously injected within 2 h, and 400 mg/m^2^ of calcium folinate (Jiangsu Hengrui Pharmaceutical Co., Ltd.) was intravenously injected within 2 h, followed 5-FU (Shanghai Xudong Haipu Pharmaceutical Co., Ltd.) at 400 mg/m^2^ was injected intravenously, and then, 2.4 mg/m^2^ of 5-FU was pumped intravenously within 46 h, 2 weeks/time. The first dose of cetuximab (Merck KGaA) was 400 mg/m^2^, intravenous infusion was completed within 2 h, and then 250 mg/m^2^ every week, intravenous infusion was completed within 1 h, once a week.

#### 2.2.2. Observation Group

Simvastatin (Chengdu Hengrui Pharmaceutical Co., Ltd.) was given on the basis of the control group, 10 mg/time, taken at night. Regularly check the patient's cholesterol level. When the total cholesterol level is ≤3.6 mmol/L or the low-density lipoprotein level is ≤ 1.94 mmol/L, consider reducing the simvastatin dose for a total of 2 months of treatment.

### 2.3. Observation Index

#### 2.3.1. Efficacy Evaluation

After the treatment, the tumor size changes were observed according to CT or MRI, and the grading was performed according to the WHO efficacy evaluation standard [16], and the efficacy evaluation was performed, as given in Table 2.

#### 2.3.2. Adverse Reactions

During the follow-up, the adverse reactions of the two groups of patients were recorded, such as skin rash, diarrhea, nausea and vomiting, thrombocytopenia, leukocyte decline, and sensory neurotoxicity.

#### 2.3.3. Follow-Up

We made telephone interviews or regular review and recorded the overall survival rate of patients until March 2020.

#### 2.3.4. Analysis of Prognostic Factors

The study collected patients' age, gender, tumor location, pathological grade, peritoneal metastasis, and chemotherapy regimen and analyzed its influence on the prognosis and survival of CRC patients.

### 2.4. Statistical Analysis

The results of this experiment were statistically analyzed by SPSS 20.0 (SPSS Co., Ltd., Chicago, USA). Normally distributed measurement data are represented by (mean ± standard deviation), and the *t*-test was used for their comparison between groups. Nonnormally distributed measurement data are represented by the median (25th percentile, 75th percentile) (M (P25, P75)), and the Mann–Whitney *U* test is used for analysis. Count data were expressed by (rate), and the chi-square test was used for their comparison between groups. The Kaplan–Meier survival curve was used to analyze the difference of postoperative survival between two different treatment methods, and the log-rank test was used for comparison. Multivariate analysis adopts the multiple logistic regression model. *P* < 0.05 indicates that the difference is statistically significant.

## 3. Results

### 3.1. Comparison of Short-Term Efficacy between the Two Groups

The results showed that in the control group, 12 cases of PD, 30 cases of SD, 15 cases of PR, and 1 case of CR, ORR was 27.59% (16/58) and DCR was 79.31% (46/58). In the observation group, 4 cases of PD, 24 cases of SD, 27 cases of PR, and 3 cases of CR, ORR was 51.72% (30/58) and DCR was 93.10% (54/58). ORR and DCR in the observation group were higher than those in the control group (*P* < 0.05), as shown in Figure 1.

### 3.2. Comparison of Adverse Reactions between the Two Groups

During the follow-up, the control group had 7 cases of rash, 6 cases of diarrhea, 11 cases of nausea and vomiting, 3 cases of platelet decline, 7 cases of white blood cell decline, and 5 cases of sensory neurotoxicity, and the total incidence of adverse reactions was 67.24% (39/58). In the observation group, there were 4 cases of rash, 4 cases of diarrhea, 7 cases of nausea and vomiting, 2 cases of platelet decline, 5 cases of white blood cell decline, and 3 cases of sensory neurotoxicity, and the total incidence of complications was 43.10% (25/58), and the total incidence of adverse reactions in the observation group was lower than that in the control group (*P* < 0.05), as shown in Figure 2.

### 3.3. Comparison of Overall Survival between the Two Groups

The results showed that the survival rates of the control group within 1, 3, and 5 years were 53.45% (31/58), 32.76% (19/58), and 18.97% (11/58), respectively. The survival rates within 1, 3, and 5 years of the observation group were 72.41% (42/58), 51.72% (30/58), and 37.93% (22/58), respectively. The survival rates of the observation group in 1, 3, and 5 years were higher than those in the control group (*P* < 0.05). The median survival time of the observation group was 38 months, and the median survival time of the control group was 25 months. The median survival time of the observation group was higher than that of the control group, and the log-rank test was *P*=0.007, as given in Table 3 and Figure 3.

### 3.4. Univariate Analysis of Mean Prognosis Survival Time in CRC Patients

Univariate analysis showed that the average survival time of CRC patients had nothing to do with age, gender, and tumor location (*P* > 0.05). Pathological grade, peritoneal metastasis, and chemotherapy regimen were associated with the mean survival time of CRC patients (*P* < 0.05), as given in Table 4.

### 3.5. Multivariate Analysis of the Mean Prognosis Survival Time of CRC Patients

Multivariate logistic analysis showed that pathological grade and peritoneal metastasis were risk factors affecting the mean survival time of CRC patients (*P* < 0.05). The results are given in Tables 5 and 6.

## 4. Discussion

In the global incidence of malignant tumors, CRC ranks the third, second only to lung cancer and stomach cancer. As a common gastrointestinal malignant tumor, CRC lacks specific symptoms at the early stage of onset, so most patients are already in the middle and late stages when diagnosed [17, 18]. The mFOLFOX6 is a standardized regimen for the treatment of advanced CRC, in which oxaliplatin and 5-FU are the main drugs that play a role [19, 20]. Oxaliplatin is a novel platinum-based anticancer drug that can inhibit DNA replication and transcription by targeting DNA. By inhibiting thymidylate synthase activity, 5-FU can make tumor cells stay in the S phase, thus exerting its antitumor effect [21, 22].

K-RAS is a protooncogene that plays a controlling role in cell growth and differentiation mechanisms. Some carcinogens convert it into active oncogenes through point mutations. K-RAS mutations occur on exons 2, 3, and 4, and exon 2 is a common mutation site for K-RAS mutations. The mutation of K-RAS gene is a common oncogene in CRC, and the incidence of mutation in Asians is 29–62.9% [23, 24]. Various genes, such as EGFR and K-RAS, are involved in the occurrence of CRC. K-RAS is a key gene in the EGFR signaling pathway. By encoding RAS protein, EGFR signals are transmitted to mitogen-activated protein kinases (MAPKs), which are involved in the regulation of cell growth, proliferation, differentiation, and angiogenesis [25, 26]. Cetuximab is a monoclonal antibody that acts as a molecular targeted tumor drug, targeting EGFR, competitively binding to the extracellular domain of EGFR with the epidermal growth factor, blocking signal transduction, and thereby inhibiting the proliferation of cancer cells [27, 28]. Studies have found that K-RAS gene is a key molecule in the EGFR signaling pathway, which can encode and strictly regulate RAS protein. Cetuximab can effectively block its signal transduction, thus inhibiting tumor growth. Therefore, cetuximab has significant efficacy in patients with wild type of K-RAS gene [29]. When K-RAS mutations occur, the RAS protein continues to activate, resulting in continued activation of the signaling pathway, and the targeting EGFR inhibitor loses its inhibitory effect on tumor cell growth, so patients with K-RAS mutations do not benefit from cetuximab therapy. Simvastatin is a 3-hydroxy-3-methylglutarate monoacyl-CoA (HCG-CoA) reductase inhibitor, which can not only play its role in lowering blood lipid in cardiovascular diseases but also participate in cell proliferation and apoptosis. Simvastatin can increase the sensitivity of K-RAS mutant CRC cells to cetuximab, thereby inhibiting cell proliferation. In addition, simvastatin can inhibit the innate growth pathway of cells by upregulating the expression of the preapoptotic protein Bad and downregulating the expression of the antiapoptotic protein Bcl-xl. Combined application of simvastatin and cetuximab can promote the apoptosis of K-RAS mutant CRC cells and reverse their drug resistance [30–32].

The results of this study showed that in the control group, 12 cases of PD, 30 cases of SD, 15 cases of PR, and 1 case of CR, ORR was 27.59% (16/58) and DCR was 79.31% (46/58). In the observation group, 4 cases of PD, 24 cases of SD, 27 cases of PR, and 3 cases of CR, ORR was 51.72% (30/58) and DCR was 93.10% (54/58). ORR and DCR in the observation group were higher than those in the control group. During follow-up, in the control group, there were 7 cases of rash, 6 cases of diarrhea, 11 cases of nausea and vomiting, 3 cases of thrombocytopenia, 7 cases of leukocyte descent, and 5 cases of sensory neurotoxicity, and the total incidence of complications was 67.24% (39/58). In the observation group, there were 4 cases of rash, 4 cases of diarrhea, 7 cases of nausea and vomiting, 2 cases of thrombocytopenia, 5 cases of leukopenia, and 3 cases of sensory neurotoxicity, and the total incidence of complications was 43.10% (25/58). The incidence of adverse reactions in the observation group was lower than that in the control group. These results indicate that the addition of simvastatin can improve the efficacy of CRC patients and reduce the total incidence of adverse reactions. The reason was that the addition of simvastatin could reverse the resistance of CRC patients with K-RAS gene mutation to cetuximab and alleviate the chance of adverse reactions in patients. With simvastatin and cetuximab treatment of CRC cells at the same time, the proliferation, migration, and invasion ability of tumor cells decreased, while the apoptosis rate increased. Further study on the mechanism found that simvastatin can inhibit the expression of murine sarcomatoid oncogene homologous B1 (BRAF), phosphorylated extracellular regulatory protein kinase 1/2 (p-ERK 1/2), and other proteins, thereby inhibiting the MAPKs pathway activity and reducing the resistance of CRC to cetuximab [33].

The results of this study showed that the 1st, 3rd, and 5th year survival rates of the control group were 53.45% (31/58), 32.76% (19/58), and 18.97% (11/58.), respectively. The 1st, 3rd, and 5th year survival rates of the observation group were 72.41% (42/58), 51.72% (30/58), and 37.93% (22/58), respectively. The survival rates at 1, 3, and 5 years in the observation group were higher than those in the control group. The median survival time of the observation group was 38 months, and the median survival time of the control group was 25 months. The median survival time of the observation group was higher than that of the control group. It shows that the addition of simvastatin can increase the sensitivity of CRC patients with K-RAS gene mutation to cetuximab and delay the progression of the tumor. This may be related to the expression of simvastatin-induced apoptosis-related proteins.

The univariate analysis results of this study showed that the average survival time of CRC patients has nothing to do with age, gender, and tumor location. Pathological grade, presence or absence of peritoneal metastasis, and chemotherapy regimens are related to the average survival time of CRC patients. Multivariate logistic analysis showed that pathological grade and peritoneal metastasis are risk factors that affect the average survival of CRC patients. Peritoneal metastasis is the most common site of CRC and is the second leading cause of death from CRC. The main ways of peritoneal metastasis in CRC patients are as follows. After breaking through the serous membrane, the tumor cells fell off into the abdominal cavity and were planted in the abdominal cavity for further growth. The implantation of tumor cells in the abdominal cavity can be caused by the flow of blood and lymph into the abdominal cavity by the severed blood vessels and lymphangioma embolus, the pulling and squeezing of tumor tissues during the operation, or the inflow of tumor cells through the intestinal stump with intestinal fluid. Patients with peritoneal metastasis had a worse prognosis than those without, and the higher the degree of peritoneal metastasis, the shorter the survival time [34, 35]. The addition of simvastatin is not a factor affecting the mean survival time of CRC patients, but it can prolong the overall survival time of patients within 3–5 years, and it is expected to be used as a routine drug regimen to optimize the prognosis of CRC patients.

## 5. Conclusion

The addition of simvastatin on the basis of conventional mFOLFOX6 regimen combined with cetuximab chemotherapy can effectively improve the efficacy, reduce the overall incidence of adverse reactions, improve the overall survival rate of patients, and prolong the overall survival time of patients. The study also found that pathological grade and peritoneal metastasis are the factors that affect the mean survival time of CRC patients.

## Figures and Tables

**Figure 1:** Comparison of short-term efficacy between the two groups. Note: compared with the control group, ^*∗*^*P* < 0.05.

**Figure 2:** Comparison of adverse reactions between the two groups. Note: compared with the control group, ^*∗*^*P* < 0.05.

**Figure 3:** Analysis of differences in survival between the two groups.

**Table 1:** Comparison of general data between the two groups.

General clinical data	Control group (*n* = 58)	Observation group (*n* = 58)	*t/χ* ^2^	*P*

Age (years old)	50.06 ± 9.59	50.30 ± 9.41	0.136	0.892
Gender			0.558	0.455
Male	30	34		
Female indent	28	24		
Tumor location			0.666	0.415
Left	43	39		
Right	15	19		
Pathological grade			1.451	0.229
Moderately or highly differentiated	37	43		
Poorly differentiated	21	15		
Peritoneal metastasis			0.372	0.542
Yes	5	7		
No	53	51		

**Table 2:** Patient clinical efficacy assessment criteria.

Efficacy	Criteria

PD	Lesion growth ≥ 20%, or new lesions
SD	Lesion growth < 20%, or reduction of lesion volume < 30%, maintain time ≥ 30 d
PR	Lesion reduction ≥ 30%, maintain time ≥ 30 d
CR	The lesion disappeared completely, maintain time ≥ 30 d
ORR	(PR + CR)/58 × 100%
DCR	(SD + PR + CR)/58 × 100%

PD, progressive disease; SD, stable disease; PR, partial response; CR, complete response; ORR, overall response rate; DCR, disease control rate.

**Table 3:** Survival comparison (*n* (%)).

Group	First year	Third year	Fifth year

Control group (*n* = 58)	53.45 (31/58)	32.76 (19/58)	18.97 (11/58)
Observation group (*n* = 58)	72.41 (42/58)	51.72 (30/58)	37.93 (22/58)
*χ* ^2^	4.472	4.275	5.125
*P*	0.034	0.039	0.024

**Table 4:** Univariate analysis of mean prognosis survival time in CRC patients.

Factors	Examples	The mean survival time (month)	*t*	*P*

Age (years)				
<50	47	30.15 (25.37, 33.48)	1.572	0.119
≥50	69	28.37 (24.06, 32.22)		
Sexuality				
Male	64	29.45 (24.82, 33.06)	0.559	0.577
Female	52	30.08 (25.35, 33.53)		
Tumor location				
Left hemicolon	82	30.26 (26.57, 33.83)	1.040	0.301
Right hemicolon	34	28.97 (24.83, 32.40)		
Pathological grade				
Medium-high differentiation	80	34.75 (31.81, 37.56)	13.363	≤0.01
Poor differentiation	36	22.64 (19.10, 25.36)		
Peritoneal metastasis				
No	104	33.58 (30.42, 36.39)	7.680	≤0.01
Yes	12	23.14 (19.19, 25.42)		
Chemotherapy regimen				
mFOLFOX6 + cetuximab	58	26.77 (22.72, 30.15)	12.607	≤0.01
mFOLFOX6 + cetuximab + simvastatin	58	39.04 (39.04, 43.11)		

**Table 5:** Assignment for multivariate analysis of factors.

Factors	Variables	Assignment

Pathological grade	*X*1	Medium-high differentiation = 0; poor differentiation = 1
Peritoneal metastasis	*X*2	No = 0; yes = 1
Chemotherapy regimen	*X*3	mFOLFOX6 + cetuximab = 0; mFOLFOX6 + cetuximab + simvastatin = 1

**Table 6:** Multivariate analysis of the mean prognosis survival time of CRC patients.

Variables	*B*	SE	Walds	*P*	OR	95% CI

Pathological grade	1.447	0.502	8.309	0.014	4.250	1.368–7.526
Peritoneal metastasis	1.602	0.533	9.034	0.008	4.963	1.861–8.035
Chemotherapy regimen	−0.459	0.641	5.181	0.102	0.632	0.226–1.015

## Data Availability

The data used to support the findings of this study are available from the author upon request.
